The article "Evaluation of Hepatic Fibrosis Using Ultrasound Backscattered Radiofrequency Signals and One-Dimensional Convolutional Neural Networks" was published in 2022. Journal: Diagnostics (Basel).

# Evaluation of Hepatic Fibrosis Using Ultrasound Backscattered Radiofrequency Signals and One-Dimensional Convolutional Neural Networks

**DOI:** 10.3390/diagnostics12112833

**Published:** 2022-11-17

**Authors:** Yong Huang, Yan Zeng, Guangyu Bin, Qiying Ding, Shuicai Wu, Dar-In Tai, Po-Hsiang Tsui, Zhuhuang Zhou

**Affiliations:** 1 Department of Biomedical Engineering, Faculty of Environment and Life, Beijing University of Technology, Beijing 100124, China; 2 Department of Ultrasound, BJUT Hospital, Beijing University of Technology, Beijing 100124, China; 3 Department of Gastroenterology and Hepatology, Chang Gung Memorial Hospital at Linkou, Chang Gung University, Taoyuan 333423, Taiwan; 4 Department of Medical Imaging and Radiological Sciences, College of Medicine, Chang Gung University, Taoyuan 333323, Taiwan; 5 Institute for Radiological Research, Chang Gung University, Taoyuan 333323, Taiwan; 6 Division of Pediatric Gastroenterology, Department of Pediatrics, Chang Gung Memorial Hospital at Linkou, Taoyuan 333423, Taiwan

**Keywords:** ultrasound backscattered signal, convolutional neural network, deep learning, hepatic fibrosis, ultrasound tissue characterization

## Abstract

The early detection of hepatic fibrosis is of critical importance. Ultrasound backscattered radiofrequency signals from the liver contain abundant information about its microstructure. We proposed a method for characterizing human hepatic fibrosis using one-dimensional convolutional neural networks (CNNs) based on ultrasound backscattered signals. The proposed CNN model was composed of four one-dimensional convolutional layers, four one-dimensional max-pooling layers, and four fully connected layers. Ultrasound radiofrequency signals collected from 230 participants (F0: 23; F1: 46; F2: 51; F3: 49; F4: 61) with a 3-MHz transducer were analyzed. Liver regions of interest (ROIs) that contained most of the liver ultrasound backscattered signals were manually delineated using B-mode images reconstructed from the backscattered signals. ROI signals were normalized and augmented by using a sliding window technique. After data augmentation, the radiofrequency signal segments were divided into training sets, validation sets and test sets at a ratio of 80%:10%:10%. In the test sets, the proposed algorithm produced an area under the receive operating characteristic curve of 0.933 (accuracy: 91.30%; sensitivity: 92.00%; specificity: 90.48%), 0.997 (accuracy: 94.29%; sensitivity: 94.74%; specificity: 93.75%), 0.818 (accuracy: 75.00%; sensitivity: 69.23%; specificity: 81.82%), and 0.934 (accuracy: 91.67%; sensitivity: 88.89%; specificity: 94.44%) for diagnosis liver fibrosis stage ≥F1, ≥F2, ≥F3, and ≥F4, respectively. Experimental results indicated that the proposed deep learning algorithm based on ultrasound backscattered signals yields a satisfying performance when diagnosing hepatic fibrosis stages. The proposed method may be used as a new quantitative ultrasound approach to characterizing hepatic fibrosis.

## 1. Introduction

Hepatic fibrosis is reversible in the early stage, so early detection of it is of critical importance. The evaluation of hepatic fibrosis stages is essential for prognosis, surveillance, and treatment decisions in patients with chronic liver disease [1]. Currently, liver biopsy [2] is the gold standard for liver fibrosis assessment. However, it has some limitations. First, it is an invasive test with the possibility of severe complications [3]. In addition, biopsy specimens represent a limited area of the whole liver, and a sampling error may occur. Thus, a noninvasive detection method for liver fibrosis is highly desired. Among different medical imaging modalities, ultrasound imaging is frequently used because of its real-time performance, low cost, easy access, and absence of ionizing radiation.

B-mode ultrasound imaging is widely available for hepatic fibrosis assessment. As an important branch of machine learning [4], deep learning uses computational models to extract high-throughput features from a large amount of raw data. In recent years, the continuous improvement in computer hardware has broadened the applications of deep learning. Convectional machine learning techniques usually used hand-crafted features to train the prediction models. In contrast, deep learning techniques could automatically extract abundant features for prediction in an end-to-end way. Deep learning [5] models based on convolutional neural networks (CNNs) have been used for the analysis of B-mode ultrasound images [6,7,8,9]. Lee et al. [10] used CNNs to assess patients’ fibrosis stages by processing 13,608 B-mode images from 3446 liver fibrosis patients. Their networks obtained an accuracy of 76.4% and an area under the receive operating characteristic curve (AUC) of 0.857 on the test set. However, B-mode ultrasound imaging is limited by its qualitative nature.

A tissue can be modeled as an ensemble of scattering particles (i.e., scatterers), and the interaction of incident ultrasound waves with tissue scatterers can be characterized by the backscattered radiofrequency signals [11,12]. Compared with B-mode imaging and image post-processing strategies, ultrasound backscattered radiofrequency signals are the most original information-carriers with regard to the analyzed tissue. The correlations between backscattered signals and tissue microstructures can be utilized to identify structural alterations in tissues that are not evident on B-mode ultrasound images [11]. Ultrasound backscattered signals have been analyzed for tissue characterization or disease diagnosis [13], e.g., for the diagnosis of breasts [14] or for monitoring the response of tumors to chemotherapy [15]. Ultrasound backscattered signals are the original echo signals received by the ultrasound transducer and contain more information than conventional B-mode ultrasound images.

Recently, deep learning based on ultrasound backscattered radiofrequency signals has been investigated. Luo et al. [16] analyzed 274 cases of patients’ ultrasound backscattered signals with CNNs to assess their osteoporosis, and the performance of their algorithm is much higher than that of traditional diagnostic methods. Han et al. [17] used one-dimensional CNNs [18] to analyze 204 patients’ fatty liver signals and gained an accuracy of 96% on the test set. Nguyen et al. [1] obtained fatty liver ultrasound backscattered signals of 52 rabbits and utilized one-dimensional CNNs to extract features and implement classification with an accuracy of 74% on the test set, exceeding 59% by the support vector machine [19]. Sanabria et al. [20] conducted a comparative experiment on 31 patients’ fatty liver backscattered signals. They utilized one-dimensional, two-dimensional, and three-dimensional CNNs to analyze the different representations of signals and concluded that different representations of data have an impact on the performance of the networks. However, only 31 cases of data were involved. Cheng et al. [21] used one-dimensional bidirectional recurrent neural networks [22] to analyze 160 rats’ hepatic fibrosis backscattered signals and gained accuracies of above 83% and 80% on the training set and the test set, respectively. However, the feasibility of using ultrasound backscattered signals and deep learning to evaluate human liver fibrosis remains unknown.

In this study, we proposed a method to evaluate human liver fibrosis using ultrasound backscattered radiofrequency signals and one-dimensional CNNs. The proposed CNN models were trained and evaluated on ultrasound radiofrequency signals collected from 230 participants. Experimental results showed that the proposed method yielded a satisfying performance for diagnosing human liver fibrosis.

## 2. Materials and Methods

Figure 1 shows the algorithmic steps of the proposed method. B-mode ultrasound images were reconstructed from backscattered radiofrequency signals. The region of interest (ROI) was manually outlined to obtain the signals within the ROI, i.e., ROI signals. The data normalization technique was introduced to normalize the ROI signals, which can improve the performance and training stability of the model. Specifically, for a frame of ROI signals, *X*, the min–max normalization method was used:

(1) $$X^{\prime }=\left(X-X_{min}\right)/\left(X-X_{max}\right),$$

where *X*’ is the normalized signal, and *X_min_* and *X_max_* are the minimum and maximum values of *X*. Data augmentation [23] has been frequently used in deep learning. In this study, a data augmentation method was introduced to balance the dataset distribution of different hepatic fibrosis stages, which will be described in Section 2.2. The preprocessed signals of training sets were fed into the one-dimensional CNN to train different CNN models. The preprocessed signals of testing sets were input to the trained CNN models to predict the classification. In this study, we trained four kinds of one-dimensional CNN models corresponding to four kinds of hepatic fibrosis classification experiments: (i) ≥F1, namely binary classification of F0 vs. F1–F4; (ii) ≥F2, namely, binary classification of F0–F1 vs. F2–F4; (iii) ≥F3, namely, binary classification of F0–F2 vs. F3–F4; and (iv) ≥F4, namely, binary classification of F0–F3 vs. F4.

### 2.1. Clinical Data

Clinical ultrasound backscattered radiofrequency data of liver fibrosis, used in our previous study [24], were revisited. The data collection was approved by the Institutional Review Board of Chang Gung Memorial Hospital in Taiwan. All participants signed an informed consent form, and the experimental method was performed in accordance with the approved guidelines. A clinical ultrasound scanner (Model 3000, Terason, Burlington, MA, USA) was used to collect the ultrasound radiofrequency signals of the participants. The center frequency of the convex-array transducer was 3 MHz, and the sampling frequency was 12 MHz. Each frame of backscattered signal consisted of 256 A-lines. Each A-line contained 1247 sampling points. Liver fibrosis was semi-quantitatively evaluated using the liver biopsy and the METAVIR scoring system, which was the clinical gold standard for staging liver fibrosis: F0 = no fibrosis, F1 = portal fibrosis with no septa, F2 = portal fibrosis with few septa, F3 = bridging fibrosis with many septa, and F4 = cirrhosis (nodular stage). The METAVIR scores of F0–F4 were used as the reference standard for diagnosing the liver fibrosis stages when using the proposed method. A total of 230 cases of radiofrequency data (F0 = 23, F1 = 46, F2 = 51, F3 = 49, F4 = 61) were included in this study.

### 2.2. Data Augmentation

Data augmentation methods were introduced to solve the unbalanced data distribution problem and avoid overfitting [25] when training models. Taking ≥F1 as an example, the amount of F0 signals, *N*_0_, was far less than that of F1–F4, *N*_1_. To avoid overfitting, the scale of F0 data needed to be augmented by *N*_aug_ times to match that of F1–F4, i.e., *N*_aug_ = *N*_1_/ *N*_0_. Figure 2 shows the process of our data augmentation. The ROI was automatically set to 1100*256 (axial*lateral). We extracted signals from the ROI and used a sliding window sized 1024*256 (axial*lateral) to obtain *N*_aug_ frames of augmented radiofrequency data sized 1024*256 (axial*lateral). The window (purple window in Figure 2) was slid *N*_aug_ times in a step of (1100–1024)/*N*_aug_. One frame of radiofrequency data sized 1024*256 (axial*lateral) was taken each time, enabling us to obtain *N*_aug_ frames of augmented radiofrequency data. Note that the size 1024*256 was experimentally set. After data augmentation, the training sets, validation sets, and test sets were divided in accordance with a ratio of 80%:10%:10%.

### 2.3. Network Structure

In this study, we proposed a one-dimensional CNN algorithm for hepatic fibrosis evaluation (Figure 1). With the combination of convolutional layers and fully connected layers, our algorithm could perform feature extraction and classification simultaneously, simplifying diagnosis workflow and increasing classification efficiency.

Figure 1 shows the structure of the network, which was composed of four one-dimensional convolutional layers, four one-dimensional max-pooling layers, and four fully connected layers. Features extracted by convolutional layers and max-pooling layers were integrated into a one-dimensional feature vector, which was input into the fully connected layers to output the prediction. Unlike convolutional layers and pooling layers, fully connected layers [26] specialized in global features.

Convolutional layers employed different kinds of convolutional kernels to extract features, the surface layers for superficial features, and deep-seated layers for underlying features. Moreover, convolutional layers were skilled in generalization. Their capability was commonly referred to as translation invariance, making them excel at handling local features and freeing them from worrying about the locations of the features. This would cost less when training networks.

As a method for down-sampling, the max-pooling layers were mainly used for avoiding overfitting. Too many parameters could lead to a poor generalization ability of the networks, yet max-pooling layers were capable of decreasing parameters. In addition, max-pooling layers were also characterized by translation invariance, so they could deal with local features in cooperation with convolutional layers.

Activation functions brought in non-linearity, which contributed to a more extended hypothesis space, so networks could produce a more accurate classification. In our networks, we used Tanh [27] as the activation function. With a rather fast rate of convergence, Tanh could effectively avoid loss value vibration.

### 2.4. Network Configuration

The collected ultrasound backscattered signals were pre-processed using MATLAB 2019. Our deep learning models were trained and tested on a personal computer (PC). Our PC is equipped with Intel(R) Xeon(R) W-2104 CPU @ 3.20 GHz, Nvidia Quadro P400 GPU, and 16 GB RAM. The deep learning framework was Pytorch (version 1.11.0). In our experiments, the batch size was set to 256 and the epoch to 100. It took 50 s to run an epoch. We used Adam [28] (learning rate: 10^–3^, betas: (0.9, 0.999)) as the gradient optimizer and the cross-entropy function [29] as the loss function. Our networks had a simplified structure with only 14,692 parameters. Running one single radiofrequency signal costed about 0.55 ms. Therefore, the proposed method can be implemented for evaluating liver fibrosis in real time.

Figure 3 illustrates the prediction process by the trained one-dimensional CNN model. For a frame of test set of radiofrequency signals sized 1024*256, each of the 256 segments of signals was input into the trained CNN model, so 256 predictions were obtained. Let *n*_C_ and *n*_W_ denote the correct and wrong predictions. If the overall prediction *p* = *n*_C_/(*n*_C_ + *n*_W_) was greater than 0.5, the frame of test set was determined correctly predicted.

### 2.5. Evaluation Metrics

The performance of our algorithm for diagnosing hepatic fibrosis was evaluated using accuracy (ACC), sensitivity (SEN), specificity (SPE), the receiver operating characteristic (ROC) curve [30], and the AUC [30]. Classification results of samples were divided into four categories: (ii) True Positive (TP), namely, an outcome where the model correctly predicted the positive class; (ii) True Negative (TN), namely, an outcome where the model correctly predicted the negative class; (iii) False Positive (FP), namely, an outcome where the model incorrectly predicted the positive class; and (iv) False Negative (FN), namely, an outcome where the model incorrectly predicted the negative class.

ACC is a metric that summarizes the performance of a classification model as the number of correct predictions divided by the total number of predictions:

(2) ACC=(TP+TN)⁄(TP+TN+FP+FN).

SEN is defined as

(3) SEN=TP/(TP+FN).

SPE is defined as

(4) SPE=TN/(TN+FP).

ROC analysis is a graphical approach to analyzing the performance of a classifier. It uses a pair of statistics—true positive rate and false positive rate—to characterize the classifier’s performance. AUC measures the entire two-dimensional area underneath the entire ROC curve from (0,0) to (1,1). It provides an aggregate measure of performance across all possible classification thresholds. The higher the value of the AUC, the better the ability to perform classifications. The ROC analysis using the 95% confidence interval was performed to calculate the AUC in diagnosing each stage of hepatic fibrosis.

## 3. Results

Figure 4 shows the loss values as a function of training epochs for the training sets and validation sets. It can be seen that both the training loss and the validation loss were decreasing for increasing epochs and reached convergence when the number of epochs was equal to 100. This implied that overfitting was effectively suppressed by the proposed data augmentation method, even though the number of cases was limited.

Table 1 shows the number of training sets, validation sets, and test sets for different fibrosis stage classifications after data augmentation.

Table 2 shows the hepatic fibrosis classification performance of the proposed method on the test set. For fibrosis stage ≥F1, our algorithm obtained an AUC of 0.933 (ACC: 91.30%; SEN: 92.00%; SPE: 90.48%). For fibrosis stage ≥F2, our algorithm obtained an AUC of 0.997 (ACC: 94.29%; SEN: 94.74%; SPE: 93.75%). For fibrosis stage ≥F3, our algorithm obtained an AUC of 0.818 (ACC: 75.00%; SEN: 69.23%; SPE: 81.82%). For fibrosis stage ≥F4, our algorithm obtained an AUC of 0.934 (ACC: 91.67%; SEN: 88.89%; SPE: 94.44%). It can be seen that the proposed method yielded an improved performance compared to the networks of Han et al. [17] and Nguyen et al. [1]. Figure 5 shows the ROC curves of the four classifications of hepatic fibrosis stages. These results demonstrated that our algorithm could yield an accurate classification of hepatic fibrosis stages.

## 4. Discussion

In this study, we proposed an approach that used one-dimensional CNN models to analyze liver ultrasound backscattered signals collected from participants. By considering the radiofrequency signal as a one-dimensional signal segment, a large number of segments were extracted from 230 cases of backscattered data to train and test the deep learning networks. The algorithm showed promising performance in the test set. The ACC of our CNN model for ≥F1, ≥F2, ≥F3, and ≥F4 was 91.30%, 94.29, 75.00%, and 91.67, respectively, with an improved performance compared to the networks of Han et al. [17] and Nguyen et al. [1] (Table 2). It was demonstrated that using CNNs trained on ultrasound backscattered signals is feasible when evaluating human liver fibrosis. This may be due to the fact that ultrasound backscattered radiofrequency signals are the original information-carriers regarding the propagated tissue and CNNs can automatically extract abundant information from radiofrequency signals. However, we also observed that the performance of our algorithm on fibrosis stage ≥F3 is below the average, the exact cause of which is not yet well understood. A possible explanation is that our method could be insensitive to liver fibrosis changes between F0–F2 and F3–F4. Note that the number of training sets of ≥F3 is relatively smaller (Table 1). Except for that, our algorithm presented a better performance for diagnosing fibrosis stage ≥F1, ≥F2, and ≥F4.

It should be noted that directly classifying liver fibrosis stages into one of F0–F4 is quite challenging. We conducted corresponding experiments and found that the best average accuracy for the direct classification was only 25%. That is why we used four binary classifications in this study, i.e., ≥F1, ≥F2, ≥F3, and ≥F4.

Currently, the feasibility of using one-dimensional CNNs and ultrasound backscattered signals to evaluate human liver fibrosis stages remains unclear. Cheng et al. [21] applied bidirectional long short-term memory networks to analyze hepatic fibrosis signals from rats and then staged the severity of their liver fibrosis. Ultrasound backscattered signals were collected using the L6-15 linear array transducer with a center frequency of 12.0 MHz [21]. Cheng et al. [21] collected 160 cases of signals (F0: 16; F1: 30; F2: 34; F3: 32; F4: 48). They used 120 cases for training the model, 30 for validation, and 10 for testing. Their algorithm achieved accuracies of 80.7%, 90.0%, 89.7%, 93.3% and AUCs of 0.935, 0.949, 0.978, 0.990 on the test set for diagnosing fibrosis stage ≥F1, ≥F2, ≥F3, ≥F4, respectively. In this study, we used a convex-array transducer with a center frequency of 3 MHz, and the ultrasound backscattered signals were collected from liver fibrosis patients.

Our network was inspired by Han et al. [17] and Nguyen et al. [1]. The network of Han et al. [17] consisted of three convolutional layers, three max-pooling layers, and two fully connected layers. The network of Nguyen et al. [1] consisted of four convolutional layers, four max-pooling layers, and three fully connected layers. In accordance with our experiments, our network was set to contain four convolutional layers, four max-pooling layers, and four fully connected layers. Compared to the network of Han et al. [17], our network may extract deeper features with more convolutional layers, and the reception field may be improved by more max-pooling layers. Compared to the networks of Han et al. [17] and Nguyen et al. [1], the more fully connected layers of our network may help in improving the nonlinearity of the model. Another difference from the networks of Han et al. [17] and Nguyen et al. [1] was that we used a smaller convolutional kernel. Such a smaller kernel may reduce the amount of model parameters, and the receptive field of the CNN model may be expanded when deeper convolutional layers are used.

Compared to B-mode ultrasound images, ultrasound backscattered signals have several potential advantages. Firstly, ultrasound backscattered signals contain more information than B-mode images [31] or the envelope data. In addition, they are also less dependent on system settings and postprocessing operations, which can contribute to their high robustness. For instance, backscattered signals are not influenced by the dynamic range setting and filtering operations that affect the presentations of B-mode images. Although training the one-dimensional CNN models takes a considerable amount of time, the trained models can be run in real time to analyze new data.

A quantitative analysis of hepatic fibrosis is a challenging task due to its special pathology condition. Our study indicated that, with the powerful mapping capability of deep learning models, liver fibrosis can be quantitatively assessed by using patients’ ultrasound backscattered signals as the model input. Since the ability to process huge amounts of data was developed, deep learning has shown advantages in classification tasks [32]. In contrast to the conventional tissue characterization methods [33], there are several advantages of the proposed method. Firstly, instead of performing a qualitative analysis of liver fibrosis, deep learning methods are designed to conduct a quantitative analysis. Secondly, conventional methods are often learnt for computer-vision-based detection and characterization, which can be easily influenced by the presentation and post-processing of ultrasound images. On the contrary, the backscattered signals are the original signals before such operations as envelope detection, logarithmic compression, and scan conversion. Thirdly, deep learning models do not require the manual calculation and selection of features of the training data, but automatic extraction of the features of the data. Moreover, our networks have the characteristics of a simplified structure, a small number of parameters, and less computational consumption.

This study has limitations. Firstly, the experimental data were acquired from a single scanner. The cross-platform generalizability of the proposed algorithm remains to be tested. Secondly, our algorithm produced a relatively worse performance for diagnosing fibrosis stage ≥F3. In future work, we would collect data from other scanners for validation of the proposed method, and try to improve the performance of ≥F3.

## 5. Conclusions

In conclusion, one-dimensional CNN models can be developed and trained to accurately identify liver fibrosis using raw ultrasound backscattered data as model input. Our preliminary results indicate that deep learning methods based on ultrasound backscattered signals are promising in the evaluation of liver fibrosis. The proposed method may serve as a new quantitative ultrasound approach to characterizing hepatic fibrosis. However, the performance of diagnosing liver fibrosis stage ≥F3 should be improved, and automatic ROI location methods should be explored in future work. Our code will be made publicly available at https://github.com/bmehuangy (accessed on 16 November 2022).

## Figures and Tables

**Figure 1:** Algorithmic steps of the proposed method. Signal preprocessing was conducted to obtain training samples of ROI signals. The preprocessed signals are fed into the CNN for model training or testing. Conv = convolution; RF = radiofrequency; ROI = region of interest; CNN = convolutional neural network.

**Figure 2:** The process of data augmentation. RF = radiofrequency; ROI = region of interest.

**Figure 3:** Prediction process by the trained one-dimensional CNN model. RF = radiofrequency; CNN = convolutional neural network.

**Figure 4:** The values of training and validation loss as a function of training epochs for fibrosis stage ≥F1 (**a**), ≥F2 (**b**), ≥F3 (**c**), ≥F4 (**d**).

**Figure 5:** ROC curves for diagnosing hepatic fibrosis ≥F1 (red), ≥F2 (blue), ≥F3 (green), and ≥F4 (purple).

**Table 1:** Number of training sets, validation sets, and test sets for different fibrosis stage classifications.

	Training Sets	Validation Sets	Test Sets
≥F1	307	46	46
≥F2	243	35	35
≥F3	189	24	24
≥F4	280	36	36

**Table 2:** Hepatic fibrosis classification performance of the proposed method on the test set, compared to the networks of Han et al. [17] and Nguyen et al. [1].

Fibrosis Stage	Model	ACC	SEN	SPE	AUC
	Ours	91.30%	92.00%	90.48%	0.933
≥F1	Han et al. [17]	89.13%	92.00%	85.71%	0.903
	Nguyen et al. [1]	86.96%	92.00%	80.95%	0.897
	Ours	94.29%	94.74%	93.75%	0.997
≥F2	Han et al. [17]	91.43%	94.74%	90.00%	0.980
	Nguyen et al. [1]	88.57%	100.00%	75.00%	0.990
	Ours	75.00%	69.23%	81.82%	0.818
≥F3	Han et al. [17]	66.67%	45.45%	84.62%	0.706
	Nguyen et al. [1]	66.67%	54.54%	76.92%	0.517
	Ours	91.67%	88.89%	94.44%	0.934
≥F4	Han et al. [17]	88.89%	77.78%	100.00%	0.892
	Nguyen et al. [1]	86.11%	88.89%	83.33%	0.880

## Data Availability

The ultrasound radiofrequency data and the ROI masks may be provided upon reasonable requests for scientific research purposes.
